The article "Metabolic Glycoengineering: A Promising Strategy to Remodel Microenvironments for Regenerative Therapy" was published in 2023. Journal: Stem Cells Int.

# Metabolic Glycoengineering: A Promising Strategy to Remodel Microenvironments for Regenerative Therapy

**DOI:** 10.1155/2023/1655750

**Published:** 2023-02-13

**Authors:** Yi Li, Yuang Zhang, Yiqin Tao, Xianpeng Huang, Chao Yu, Haibin Xu, Jiangjie Chen, Kaishun Xia, Kesi Shi, Yongxiang Zhang, Jingkai Wang, Jiawei Shu, Feng Cheng, Shaoke Wang, Chengzhen Liang, Fangcai Li, Xiaopeng Zhou, Qixin Chen

**Affiliations:** ^1^Department of Orthopedics Surgery, The Second Affiliated Hospital, School of Medicine, Zhejiang University, 88 Jiefang Road, Hangzhou, Zhejiang, China; ^2^Key Laboratory of Motor System Disease Research and Precision Therapy of Zhejiang Province, Hangzhou, Zhejiang, China

## Abstract

Cell-based regenerative therapy utilizes the differentiation potential of stem cells to rejuvenate tissues. But the dynamic fate of stem cells is calling for precise control to optimize their therapeutic efficiency. Stem cell fate is regulated by specific conditions called “microenvironments.” Among the various factors in the microenvironment, the cell-surface glycan acts as a mediator of cell-matrix and cell-cell interactions and manipulates the behavior of cells. Herein, metabolic glycoengineering (MGE) is an easy but powerful technology for remodeling the structure of glycan. By presenting unnatural glycans on the surface, MGE provides us an opportunity to reshape the microenvironment and evoke desired cellular responses. In this review, we firstly focused on the determining role of glycans on cellular activity; then, we introduced how MGE influences glycosylation and subsequently affects cell fate; at last, we outlined the application of MGE in regenerative therapy, especially in the musculoskeletal system, and the future direction of MGE is discussed.

## 1. Introduction

The need to regenerate or replace impaired tissues is rising nowadays, owing to the extended lifespan and the attendant degenerative diseases, as well as trauma and tumors [1]. Exogenous stem cells provide convenience to obtain as well as broad differentiation attributes. They not only can propagate under a static state but also can be induced to differentiate towards specialized cells or tissues with proper stimuli, aiming to rejuvenate the degenerated tissues back to their normal functional state [2, 3].

But the stem cells also bring us a question: how to maximize their regenerative efficiency after transplantation? The fate of stem cells can be more dynamic than we expected including adhesion [4], migration [5], proliferation, and apoptosis [6]. Besides, the survival rate of stem cells after transplantation also remained unsatisfactory.

The cellular microenvironment can be considered as a fundamental entry point for these obstacles above, because the decision of cell fate is highly regulated by matrix mechanical cues [7], biochemical factors [8], and other manners like intercellular crosstalk [9]. Researchers have endeavored to grasp the characteristics of the cellular microenvironment, in which cell-surface modification might be an ideal approach to regulate it.

In general, the cell membrane provides a platform carrying proteins or molecules that assist cells to conduct essential signals from external stimuli. Modification of cell membrane can display heterologous proteins on the surface, thereby inducing cellular responses and regulating biological behaviors [10].

The major technologies of cell-surface modification include hydrophobic membrane insertion [11], chemical conjugation [12], liposome fusion [13], metabolic pathways [14], enzymatic modification [15], and genetic engineering [16]. Among them, genetic engineering is the most widely used approach which incorporates materials into the genome of cells and then encodes target receptors onto the surface, such as cargocytes [17] and chimeric antigen receptor (CAR) T cells [18, 19].

Although genetic engineering could be a robust strategy to modify membranes, it is also associated with some drawbacks: (1) the process is time-consuming; (2) genetic transfection using viral vectors may cause unpredictable risks; (3) the irreversible modification may raise safety concerns for clinical applications; (4) moreover, not all cell types can adapt to genetic alteration without side effects, particularly in stem cells [20, 21].

In contrast, metabolic glycoengineering (MGE) is a safe and reversible strategy for membrane modification using nongenetic methods. Unlike nucleic acid or proteins, the cell-surface glycans are not directly encoded by genes. Biosynthesis of glycans (glycosylation) is determined by intra- or extracellular factors such as substrate transferases, signal transduction, and metabolic pathways [22, 23]. MGE technique is aimed at manipulating glycosylation and cellular metabolism to increase the expression levels of natural glycans and, more importantly, to install nonnatural monosaccharides into cell-surface glycoconjugates, such as ketone-, azide-, thiol-, or alkyne-modified glycans [24, 25].

Since MGE exploits the inherent natural metabolic pathway of cells, the process of modification barely interferes with other cellular functions—sort of like “silent” labeling [26]. Meanwhile, the MGE strategy also has other advantages as (1) easy but efficient process by simply coculturing cells with metabolic precursors; (2) exhibits noncytotoxicity even under high concentration of treatment; (3) applicable to almost all cell types; (4) nonpermanent modification that allows controlled reversal; and (5) the diversity of sugar analogs and bioorthogonal click chemistry endows MGE with numerous choices for membrane modification.

Therefore, by modifying surface glycans' structure or expression flux to decorate the cell membrane, MGE can circumvent the limitations associated with other strategies like genetic engineering.

In this review, (1) we firstly illustrated the significant role of cell-surface glycans in cell microenvironments; (2) then, we described how metabolic glycoengineering (MGE) influences cellular behaviors, and we exemplified MGE's effect on cell fate control; (3) finally, we outlined the application of MGE in regenerative medicine with a focus on the musculoskeletal system, and the future direction is also discussed.

## 2. Cellular Microenvironment, Extracellular Matrix, and Cell-Surface Glycans

### 2.1. Microenvironment and Extracellular Matrix: Shelters for Cells

Cell microenvironments are small zones around cells that can be defined as the intercellular substance containing dynamic body fluid components [27]. Particularly, stem cells are residing in specialized microenvironments that donated as “stem cell niches,” which provide stem cells with static status and low-energy-consuming conditions to maintain their balance between self-renewal and differentiation [28].

The cell microenvironments consist of a set of elements that influence cellular activities (Figure 1), which can be mainly classified into the following types: extracellular matrix (ECM), adjacent cells (both homotypic or heterotypic), mechanical forces, proteolytic enzyme factors, and inflammatory cytokines [29]. And ECM represents the major component of the stem cell niche.

On the one hand, ECM provides cells with physical support, cytoskeletal structure, and transduction of physiological signals. The ECM components such as glycosaminoglycans (GAG) and adhesive molecules are maintaining the stability of cells, and the proper adhesion to ECM is essential for the survival of adjacent cells [30]. Partial geometric control of cell growth by spreading is also a basic mechanism for the developmental modulation of ECM [31].

On the other hand, microenvironments are rather dynamic than stuck in a rut. Cells remodel their microenvironments by altering the secretion of ECM components. Each kind of tissue creates a unique ECM composition, which is responsible for tissue-specific behaviors. The high affinity between stem cells and ECM can selectively influence the cell differentiation towards specific orientations, according to respective ECM components [32, 33] (e.g., fibroblasts to fibronectin, chondrocytes to type II collagen, or endothelial cells to laminin).

Conversely, without effective adhesion to ECM, cells tend to start the procedure of cell death such as apoptosis and necroptosis [34]. This phenomenon was initially reported in epithelial cells that the disrupted cell-matrix interaction will result in cell anoikis (a special type of apoptosis) [35]. However, the loss of function of the anoikis signals will also lead to another polarization, cancerous differentiation and metastasis [36], which reminds us about the injection of embryonic stem cells (ESCs) that generally results in teratoma formation [37].

Henceforth, considering the pluripotent of stem cells, it is critical to ensure desired interactions between cells and ECM. There could be many variations that we can precisely control for altering the specific characteristics of the microenvironment. And cell-surface glycan could be a major participant since sugars are ubiquitously present in all classes of cells, where they function as sources of energy, regulators of signaling, and participants of metabolic activity.

### 2.2. Cell-Surface Glycans: The Active Determinants of Microenvironment and Stem Cell Fate

Cellular glycans can be found in proteoglycans, glycoproteins, and glycolipids. Among all these glycoconjugates, cell-surface glycans (also called glycocalyx) are polysaccharides wrapping around the surfaces of all mammalian cells and participating in cell-cell [38] and cell-matrix [39] interactions (Figure 1). Like correspondences, these interactions mark the function of a cell, specify how it communicates with its surroundings, and also influence immune response [40].

Glycosylation, the covalent attachment of glycans, is the most abundant posttranscriptional modification of proteins in nature [41]. O-Glycosylation and N-glycosylation are two major versions of protein glycosylation. O-Glycosylation involves the attachment of monosaccharides (N-acetylglucosamine) or polysaccharides (glycans) to threonine, serine, or tyrosine, while N-glycosylation added glycans to asparagine residues selectively [42]. Consequently, differences in structural composition conferred diversity of function to different glycosylated proteins.

For example, *α*-2-6-sialylated N-glycans, but not O-glycans, could be used as markers of the differential potential of mesenchymal stem cells [43]. Cell-surface N-glycans were also proved to influence the electrophysiological properties and differential fate of neural progenitor cells [44]. Moreover, the defect in glycosylation will lead to the disrupted adhesion of epithelial cells and then impair the cellular microenvironment [45]. The glycosylation can also influence cell fate directly. For example, both N- and O-glycosylation in cells functionally modulate the early steps of osteogenic differentiation of skeletal progenitor cells [46, 47].

Among the many glycosylation processes, sialylation is a significant one that happens on the terminal of mucin protein, mediated by sialyltransferases (ST) [48]. And cellular sialylation is essential in cell adhesion because the expression of integrin ligands is closely related to it [49, 50]. Integrin determines which ECM component cells would bind to during cell development and thus selectively affects the cell morphology [51]. Beyond integrins, the selectin family is another determinant cluster of adhesion that recognizes sialylation, while the sialylated Lewis X (sLeX) is the ligand for selectin [52, 53]. And some sialylated molecules also perform direct effects on the nervous system, with some gangliosides (GM3 and GD3) that control the early development by impacting cell growth and apoptosis [54]. Moreover, the precursors of sialyation were reported to act as signaling molecules that control the differentiation of neural cells [55]. In short, the function, stability, and metabolism of glycoproteins are dependent upon correct sialylation.

Cell-surface glycans are important factors that facilitate communication with the ECM and mediate signaling cascades and, consequently, make glycosylation or sialylation an active determinant in the microenvironment, regulating cell fate in both direct and indirect manners.

## 3. Metabolic Glycoengineering: A “Silent” Method for Glycan Modification

The synthesis of cell-surface glycans is determined by substrate transferases and metabolic conditions. Herein, metabolic glycoengineering (MGE) is a nongenetic strategy for glycan modification based on metabolic precursors.

### 3.1. Overview of MGE

The main purpose of MGE is to increase the expression levels of natural glycans and install nonnatural monosaccharides into cell-surface glycoconjugates [24]. To put it in another way, MGE introduces various chemical groups into cellular glycan by artificially modified monosaccharides that bear unnatural functionalities (R-groups). While being incubated with mammalian cells, those monosaccharides can intercept the glycosylation pathways in cells, resulting in the submission of R-group-modified glycans on cell surfaces or secreted as glycoconjugate [56, 57].

Sialic acid, also known as neuraminic acid, is mainly located at the ends of the side chains of cell membrane glycoproteins, where it participates in numerous interactions between cell and microenvironment [25].

N-Acetylneuraminic acid (Neu5Ac) is the most common form of sialic acid in human cells while the N-acetyl-D-mannosamine (ManNAc) acts as the physiological precursor of all sialic acids. After ManNAc is absorbed into a cell as a precursor, it is converted to Neu5Ac with the help of specific sialyltransferases and will eventually be anchored to the residues of cell-surface sialic acid (Figure 2(a)).

The sialic acid pathway was the first glycosylation pathway to be utilized in MGE [58], and it is also the most commonly used pathway nowadays. The reason why the sialic acid pathway becomes a suitable choice for MGE is relevant to the remarkable substrate promiscuity of sialyltransferases [59, 60], which provides the possibility for the modified analogs to successfully intercept glycosylation pathways, resulting in the chemically modified sialic acid (Figure 2(a)). For example, N-propionyl-mannosamine (ManNProp) is an analog of ManNAc with a propionyl group on the N-acyl side chain (Figure 2(b)Ba), and the metabolism of ManNProp eventually submits N-propionyl-neuraminic acid (Neu5Prop) on the cell membrane surface [61].

### 3.2. Metabolic Precursors of Sialic Acid

Since Kayser et al. developed the 1^st^ generation of ManNAc analogs (ManNProp, ManNBut, and ManNPent) in the 1990s [56], more than dozens of unnatural monosaccharides have been synthesized as appropriate precursors for MGE. Among all these ManNAc analogs, two major categories can be grouped: (i) aliphatic analogs and (ii) bioorthogonal analogs.

Aliphatic analogs are characterized by their N-acyl side chains which elongated with one or more methylene groups. Slight modifications of the sialic acid N-acyl side chain, such as the introduction of hydrophobic methylene, will cause significant impacts on specific cell-surface biological functionalities (Figure 2(b)Ba), including virus infection receptors [62], cell-surface differentiation markers [63], and cell proliferating regulation [64]. Thus, MGE based on aliphatic ManNAc analogs is aimed at bringing additional biological features to cells and then consequently influencing their behavior and fate.

Bioorthogonal analogs are synthesized with N-acyl side chains carrying reactive R-groups which are absent in biological systems but could be utilized for further chemical conjugations or reactions (Figure 2(b)Bb). Bioorthogonal chemistry enables the installation of artificial functionalities onto the cell surface, such as drugs [65], ligands [66], macromolecules [67], or fluorescent dyes [68]. For example, azide-functionalized N-acetylmannosamine (ManNAz) can produce azide groups on N-acyl side chains of sialic acid. Azide groups are absent from mammalian cells, but it holds bioorthogonal reactivity with most biofunctional groups. To be specific, based on the high efficiency of reactions between dibenzocyclooctyne (DBCO) and azide groups, certain DBCO-modified substances can be attached to these azide groups on cell surface, resulting in the combination that we expected. Theoretically, any functional substance of our interests can be installed onto sialic acid by using the two-step bioorthogonal reaction. This connecting process undergoes copper-free click chemistry, which is characterized by its linkage stability, biocompatibility, and noncytotoxicity.

Beyond sialic acid, other glycosylation pathways have also been exploited with the development of MGE, such as L-fucose [69], GlcNAc (N-acetylglucosamine) [70], and GalNAc (N-acetylgalactosamine) [71], which provide more opportunities for MGE's application in various fields. A comprehensive description of MGE can be seen in these review articles [26, 72, 73]. But the major effort in MGE continued to concentrate on the sialic acid pathway, due to its biological importance and the outstanding permissibility of sialyltransferases for nonnatural analogs.

In the next section, we will focus our sight on applications of MGE in inducing biological cellular response, particularly in cell fate control.

## 4. The Impact of MGE on Cell Fate

Considering the significance of glycocalyx in biological activities as well as the accessibility of sialic acid to be chemically modified, glycans can act as targets for controlling cell fate.

Evidence is adequate that sialic acid precursors can precisely influence cellular behaviors. For example, ManNBut could reversibly inhibit the expression of cell-surface polysialic acid (polySia) while ManNProp did not downregulate it, due to the shorter N-acyl side chain of ManNProp [74]. ManNProp and ManNBut only differ from 1 methylene unit (-CH3) in their terminal structure of the N-acyl side chain (Figure 2(b)Ba), but these two analogs tend to elicit different biological consequences.

Hence, in this section, we will summarize current approaches and applications of MGE analogs in modulating cell biological behaviors, including adhesion, differentiation, migration, homing, survival, and secretion, and the related mechanism is also summed up.

### 4.1. Adhesion

Different chemical functional groups assembled on the surface can induce cell adhesion, and the strongest effect comes from methylene [75]. In 2002, Villavicencio-Lorini et al. reported that ManNProp stimulated the upregulation of intracellular *β*1-integrin receptors and eventually resulted in stronger adhesion between fibronectin and HL60 cells (the leukemia cell line) [76]. Although both natural and unnatural precursors of sialic acid can induce the upregulation of *β*1-integrins, the expression level induced by ManNProp (nonnatural) was twice than that of ManNAc (natural).

For the lack of the key enzyme of sialic acid pathway, HL60 cells do not express any sialylated molecules under normal conditions. But by incorporating Neu5Prop (Figure 2(a)) onto the glycans of HL60 cells, ManNProp dramatically increased the sialyl Lewis X (sLeX) biosynthesis, resulting in the promoted adhesion between HL60 cells and selectins [52]. The same effect of sLeX increasing was also detected in ManNProp-treated mesenchymal stromal cells (MSCs), which have been shown to target MSCs to bone marrow [77, 78].

Furthermore, the half-life time of some glycoproteins is modulated by terminal sialic acid. Thus, by altering the metabolic flux of sialic acid, MGE not only changes the glycan structure on the cell surface but can also affect the biostability of certain proteins. For example, ManNProp treatment extended the half-life of the sialylated molecule (CEACAM1) from 26 hours to 40 hours, which mediates cell-cell adhesion in PC12 cells (the rat pheochromocytoma cell line) [79].

Apart from methylene (-CH3), thiol is another kind of functionality that can promote cell adhesion.

Ac5ManNTGc is the hyperacetylated ManNAc analog with a thiol group on its N-acyl side chain (Figure 2(b)Bc). Jurkat cell is a T-lymphoma-derived cell line which possesses no adhesive property, but Ac5ManNTGc can incorporate thiols into the nonadhesive Jurkat cells [80] and then stimulate the additional cell adhesion to maleimide-functionalized surfaces [81]. These modified Jurkat cells also clustered spontaneously to produce numerous ECM components and upregulate their expression of *β*1-integrin, MMP-9, and CD44, which are involved in their attachment to ECM during T-lymphoma metastasis [82].

In these seminal explorations above, researchers generally use aliphatic analogs to modify membrane and elicit direct cell adhesion. But recently, bioorthogonal analogs (Figure 2(b)Bb) are also being exploited to enhance artificial adhesion since the click chemistry could endow cells to be chemically connected, building the “functional cell complexes.” For example, Ac4ManNAz introduces azide groups into the cell surface as the first step; secondly, those azide groups are modified, respectively, with tetrazine (Tz) or *trans*-cyclooctene (TCO); thirdly, by mixing the modified cells, Tz-TCO click chemistry could produce intercellular adhesion [83, 84]. Click reaction between cyclodextrins (CDs) and adamantly (Adam) was also used to artificially combine A459 lung tumor cells and Jurkat cells, then triggered the activation of NK cells, and leads to the death of cancer cells [85].

In summary, the adhesion of cells to their microenvironment is indispensable because a cell cannot survive in the manner of an individual [3]. Because sialic acid participates in cell-cell and cell-matrix adhesion, it is worth wondering whether MGE can decide cell fate by introducing nonnatural glycans.

### 4.2. Differentiation and Proliferation

The earliest application of metabolic glycoengineering in regenerative medicine was conducted in neural cells by Schmidt et al. in 1998. ManNProp incubation in neural progenitor cells (NPC) induced the proliferation of astrocytes, microglia, and early-stage oligodendrocytes [86]. Buttner et al. also reported that ManNProp stimulated axonal outgrowth both in neuron cells and PC12 cells [87].

It has been demonstrated that ManNProp increased the calcium fluctuation in these cells [88]. Likewise, the adhesion effect of ManNProp in HL60 cells was also caused by intracellular calcium spiking, which thereby promoted the cell marker of monocytic differentiation [89]. And systemic administration of ManNProp significantly increased the axonal regeneration after sciatic nerves were transplanted into the mouse model [90], which proved to depend on the polysialyltransferase activity in the nerve graft [91].

It was suggested for the first time that ManNAc analogs can directly influence proliferation and axonal growth, and it is worth exploring for their influence on differentiation.

As described in Section 4.1, Ac5ManNTGc endows Jurkat cells with adhesive properties by introducing thiols. Moreover, when being applied in the human embryoid body–derived (hEBD) stem cells, Ac5ManNTGc was proved to stimulate neural lineage differentiation in the absence of Wnt signaling proteins [81], which are usually indispensable for neural differentiation [92].

In contrast, those cells treated with Ac5ManNGc—which lacks thiol—showed only slight changes in the cytoskeleton, indicating no influence on differentiation. It can be inferred that the thiol group of the ManNAc analog is the key factor in enhancing cell adhesion and neural differentiation. But the upregulation of Wnt signal was only found on a gold-covered surface, indicating that the high-affinity bond of thiols was confined to the complementary scaffolds.

Du et al.'s group recently synthesized two novel thiol analogs—Ac5ManNTProp and Ac5ManNTBut (Figure 2(b)Bc)—which are claimed to install thiol on an elongated N-acyl side chain, thereby enhancing the ability of glycans to interact with other thiols, and overcome the necessity for complementary scaffolds [93]. When treated with human neural stem cells (hNSCs) and human adipose-derived stem cells (hADSCs), respectively, the stronger morphological responses were observed with Ac5ManNTBut, while Ac5ManNTProp exhibited better biocompatibility.

Among the thiol-treated hNSCs, the apparent neural differentiation was found as well as the upregulation of the Wnt signaling pathway. It was also demonstrated that the longer the N-acyl side chains were, the stronger the activation of Wnt signaling would be—raising from Ac5ManNTGc to Ac5ManNTProp and the strongest up to Ac5ManNTBut. According to the fact that the Wnt signaling also hinders adipogenesis [94], both Ac5ManNTProp and Ac5ManNTBut did inhibit the adipocyte differentiation in hADSCs [93]. The biosafety and scaffold-independent properties will make those ManNAc analogs be attractive tools in neural regenerative medicine.

In the previous studies, thiol-modified ManNAc analogs were usually used as bioorthogonal handles to link drugs to antibodies through maleimide conjugation [95]. But the work of Yarema et al. demonstrated that bioorthogonal analogs may also induce direct biological responses similar to those aliphatic analogs. And the outcome of thiol modification could be changed by altering the length of the aliphatic side chain.

By introducing topological cues in the growth substrate and creating the glycoengineered binding interface, cell adhesion can be enhanced, gene expression can be regulated, and thus cell fate can be controlled, where the chemical composition of the cell surface is altered to promote carbohydrate-mediated interaction.

### 4.3. Migration and Homing

Beyond differentiation, cell migration and homing are regarded as the other two important activities that associated with sialic acid.

For instance, tumor cells usually synthesize polysialic acid (polySia) to regulate their ECM adhesion and migrate properties thereby becoming more metastatic [96]. Nagasundaram et al. reported a remarkable reduction of polySia in MCF7 breast cancer cells when treated with a series of ManNAc analogs (ManNProp, ManNBut, and ManNPent). Furthermore, the decreased level of natural polySia significantly suppressed adhesion and then inhibited breast cancer migration [97].

Conversely, compared with cancer cells, stem cells showed opposite responses. Incubation of ManNProp endows MSCs with a high expression level of sLeX which enhanced their osteotropism, also known as “homing” [77]. This homing effect of MSCs is determined by the interaction between sLeX and selectins, which is also involved in the neurotropism of NSCs [98].

In addition, supplementation with 3F-Neu5Ac was proved to increase migration and adhesion of MSCs and then promoted their survival rate in an ischemia model [63]. And the inhibition of osteogenic and adipogenic differentiation was also observed in those MSCs treated with 3F-Neu5Ac.

### 4.4. Apoptosis, Survival, and Secretion

The fact that sialic acid metabolism participates in cell apoptosis [54, 99] is also reflected in ManNAc analogs. By modulating metabolic flux of the sialic acid pathway, ManNAc analogs have the potential to either amplify or reduce cell apoptosis.

Research by Kim et al. demonstrated that ManNAc analogs can modulate cell apoptosis directly through N-acyl group effects, or indirectly via hydroxyl group effects. Especially, the ketone-bearing analog (Ac4ManNLev) possesses strong toxicity via inhibiting the sialic acid pathway [100]. Furthermore, the combination of 3,4,6-O-tributanoylation with the ManNLev (3,4,6-O-Bu3ManNLev) resulted in the most apoptotic ManNAc analog, which thus being a promising anticancer drug candidate [101]. Instead, 1,3,4-O-Bu3ManNAc increased the sialylation level of SW1990 cells (pancreatic cancer cells) up to 2-fold and in essence resensitize the SW1990 cells to anticancer drugs [102].

While the ketone groups are used to induce cell apoptosis, azide groups are promising in enhancing the survival rate of those cells seeded in biomaterials. Mao et al. fabricated DBCO-modified polymers as an MGE responsive platform and obtained azide-labeled macrophages through Ac4ManNAz. The bioorthogonal reaction between DBCO and azide accomplished fast in situ cellularizations and dramatically increased the selective capture and survival rate of the macrophages in the DBCO-modified scaffold [103].

Another intriguing application is the single-cell encapsulation via MGE. Oh et al. [104] utilized DBCO-azide conjugation to wrap every neural progenitor cell (NPC) with a layer of PEG polymer. The single-cell encapsulation with optimized stiffness changed the ADCY8-cAMP pathway due to the mechanical properties of polymers and enhanced the trophic factor secretion of NPCs, which reduced the required amounts of cells for therapy.

### 4.5. Brief Summary

All in all, the sialylation of N-glycans is tightly associated with the response to microenvironmental cues. Altering the structure of cell-surface glycans by metabolic glycoengineering (MGE) will certainly affect signaling pathways, no matter of incorporating either bioorthogonal or aliphatic modification.

From the analysis of the microarray data, up to a total of 14 pathways have been proved to be modulated via MGE products [105], including apoptosis, cell adhesion molecules, cell differentiation, leukocyte migration, and Wnt signaling as well as NF-*κ*B signaling.

Taken together, these applications have established the MGE analogs as versatile tools for modulating biological activity such as cell adhesion, differentiation, migration, survival, or secretion, which may positively impact the therapeutic potential of the stem cells.

## 5. Applying MGE in Regenerative Medicine: With a Focus on Musculoskeletal System

Sialic acid possesses another name called “neuraminic acid,” since it was initially isolated from neural tissues and highly expressed in the neural system. Hence, the earliest therapeutic exploration of MGE had mostly focused on neural lineage differentiation and neural tissue regeneration.

But sialic acid is widely existing in plentiful cells and tissues, rather than exclusively in neural systems. Along with the prospering development of MGE, this carbohydrate-based strategy also showed potential in therapy for the musculoskeletal system. In this section, we will introduce the application of MGE in regenerative medicine with a focus on the intervertebral disc and cartilage, which all tend to be ideal targets for metabolic glycoengineering.

### 5.1. Chondrogenic Differentiation and Cartilage Tissue Regeneration

The inflammatory environment in osteoarthritis (OA) joints disrupts the homogenesis of the articular microenvironment, thus reducing the ability of cartilage to regenerate and limiting the efficacy of OA therapeutics. To date, some carbohydrate-based molecules have shown potential in stem cell differentiation and chondrocyte regeneration.

#### 5.1.1. Glucosamine-Metabolic Glycoengineering Produced by “Nature”

Glucosamine (GlcN), a natural sugar that widely exists in cartilage, serves as the precursor for glycosaminoglycans (GAG), which are important components of the ECM secreted by chondrocytes and help sustain the flexibility, toughness, and strength of this connective tissues [106]. Probably, we could define that glucosamine is kind of like a natural precursor of MGE since it helps with the supplement of ECM as many other analogs did.

It is well-known that GlcN has been regarded as a proper chondroprotective drug candidate for decades [107]. In 2007, Derfoul et al. demonstrated that the treatment of GlcN contributed to maintaining the chondrogenic phenotypes both in osteoarthritic chondrocytes and MSCs and promoted the secretion of ECM, as well as partially inhibited the expression of IL-1*β* and matrix metalloproteinase-13 (MMP-13) [108], which account for the clinical therapeutic effect of GlcN on OA, such as anti-inflammatory and chondroprotective.

In 2005, Khoo et al. reported the inducing effect of GlcN on the differentiation of embryonic stem cells (ESCs) [109]. By encapsulating GlcN in hydrogels, it was demonstrated that GlcN significantly enhanced the accumulation of chondrogenic ECM in the embryonic body (EB) [110]. Moreover, recent studies have shown that the treatment of GlcN also promoted the proliferation of chondrocytes via the Wnt/*β*-catenin signaling pathway [111], similar to the stem cells treated with ManNAc analogs [93].

The N-butyryl analog of glucosamine, “GlcNBut,” was also found to stimulate normal chondrocytes to secrete ECM [112]. Poustie et al. cultured the normal chondrocytes with several glucosamine analogs, including GlcNAc, GlcNBut, and GlcNProp. The treatment of GlcNBut to chondrocytes increased the level of expression of mRNA of collagen-II and aggrecan, while GlcNAc and GlcNProp had no such influences. GlcNBut showed its potential to alleviate OA disease, but whether it could be applied *in vivo* to rejuvenize the senescent cartilage remained uncertain.

#### 5.1.2. Tributanoylated GlcNAc, GalNAc, and ManNAc: The Hexosamine Analogs Derived from Short-Chain Fatty Acid

Despite the widely reported anti-inflammatory and chondrogenic differentiation properties of GlcN, its direct influence on the regeneration of cartilage had remained inconclusive for a long time [113, 114]. From a perspective of tissue engineering, the effective treatment of osteoarthritis requires a strategy that can both reduce inflammation and increase tissue production.

Among the efforts in reducing inflammation, NF-*κ*B signaling is an intriguing therapeutic target in OA disease since it regulates the expression of many inflammatory mediators and matrix-degrading enzymes [115].

As it is mentioned in Section 4.5, the NF-*κ*B signaling pathway can be modulated via MGE products [105], and the inhibition of NF-*κ*B in cancer cells was previously observed with the short-chain fatty acid- (SCFA-) modified hexosamine analogs (Figure 2(b)Bd), such as tributanoylated 3,4,6-O-Bu3ManNAc and 3,4,6-O-Bu3ManNLev [101, 116]. After cellular uptake, those tributanoylated sugars can be naturally metabolized to their downstream byproducts, for example, from 3,4,6-O-Bu3ManNAc to ManNAc with three butyrate groups. The hexosamine part acted as a “core” for the biosynthesis of glycosaminoglycans (GAG), while the butyrate moieties modulated inflammation signaling pathways.

In addition to 3,4,6-O-Bu3ManNAc, the tributanoylated GlcNAc analog (3,4,6-O-Bu3GlcNAc) downregulated the NF-*κ*B activity in those cancer studies too [116], which was reminiscent of the therapeutic effect of GlcNAc analogs in OA. And not surprisingly, the same effect of the tributanoylated GlcNAc (3,4,6-O-Bu3GlcNAc) was observed in OA chondrocytes, which promoted their ECM accumulation and inhibited inflammation [117], indicating that 3,4,6-O-Bu3GlcNAc might have the potential to reproduce cartilage tissue.

To get a comprehensive grasp of the characteristic of tributanoylated hexosamine analogs and to optimize their therapeutic effect in OA, Coburn et al. synthesized three analogs named as 3,4,6-O-Bu3GalNAc, 3,4,6-O-Bu3ManNAc, and 3,4,6-O-Bu3GlcNAc, for evaluating their effect on chondrocytes and mesenchymal stem cells, [118]. All the analogs inhibited the expression of NF-*κ*B and increased the cartilage-like ECM accumulation in OA chondrocytes, while the GalNAc-Bu3 induced the strongest responses at a concentration with negligible cytotoxicity.

The *in vivo* investigation of GalNAc-Bu3 in rat OA models by Kim et al. showed that GalNAc-Bu3 induced cartilage tissue production both in MSCs and human OA chondrocytes by regulating the Wnt/*β*-catenin signaling, the negative pathway engaged in OA same as NF-*κ*B [119]. Furthermore, GalNAc-Bu3 extended the survival of MSCs despite the rapid clearance rate of the synovial fluid.

Notably, the therapeutic effects of these tributanoylated analogs are not simply due to their catabolized metabolites, since their isomers are incapable to suppress the NF-*κ*B activity (such as 1,3,4-O-Bu3GlcNAc), suggesting that the specific location of butyrate influences those effects [117].

Taken together, the potential of hexosamine analogs derived from SCFA could be translated as suitable drug candidates for OA disease, and the prospect of MGE-based carbohydrates in inducing chondrogenic differentiation of MSCs is calling for further investigations.

### 5.2. Prospect of MGE in Intervertebral Disc Regeneration

The intervertebral disc (IVD) is comprised of nucleus pulposus (NP), annulus fibrosus (AF), and endplates (EPs), while the NP is the highly hydrated region that is located at the inner central part of IVD [120]. It is well-known that the aging and dysfunction of NP cells lead to the degeneration of NP, which is an important initial process in the pathology of intervertebral disc degeneration (IVDD) [121].

#### 5.2.1. Values and Obstacles of Stem Cells in IVDD Regeneration

Exogenous supplementation of mesenchymal stem cells (MSCs) has been proved to enhance the height and water content of the intervertebral disc [122, 123]. However, the harsh microenvironment in the degenerated NP (hypoxia, lack of blood supply, acidity, and hyperosmolality) severely hinders the survival and function of any transplanted cells [124–126].

As has been discussed earlier, the effective adhesion between stem cells and ECM can optimize cell behavior and tissue regeneration [127]. In the context of discs, it has been reported that the high affinity between MSCs and type II collagen promoted the differentiation towards NP cells and helped MSCs maintain NP-like phenotypes [128, 129]. But a proper method to ensure the adhesion between transplanted cells and ECM components *in vivo* remains unclear in IVDD therapy. Herein, the MGE technique might help.

#### 5.2.2. Enhance Nucleus Pulposus Regeneration by MGE

Based on previous studies demonstrating that modification of cell-surface glycan can modulate the adhesion property of cells [89], MGE might stimulate inner bounding to ECM that facilitates the differentiation of MSCs and then regenerate the disc.

An example from our laboratory validated that ManNProp, introducing extra -CH3 on sialic acid, greatly enhanced the adhesion ability of ADSCs, especially the selective adhesion with type II collagen [130]. Moreover, this cellular response promoted the efficiency of differentiation towards NP-like cells in a *β*1-integrin-dependent manner, by stimulating FAK/ERK pathway.

In rat IVDD models, better mechanical performance, increased water content, and the reconstruction of NP structure were observed after the transplantation of engineered cells with collagen scaffolds. It manifested that the MGE strategy not only promoted stem cells to overcome the harsh microenvironment in degenerated NP tissues but also benefits the regeneration of NP.

Designing biomaterials to improve cell adhesion is not a novel topic. However, the current efforts are mainly focusing on ECM engineering to “lure” passive adhesion by adding purified proteins and molecules [131, 132]. But the complexity of the synthetic procedure and the instability of proteins have confined the translational research of ECM modification. To address these limitations, we have highlighted the feasibility of cell membrane modification to produce “active adhesion” via glycoengineering and thus benefit disc regeneration.

Meanwhile, cartilage is an analogous connective tissue of IVD with a similar biofunction. And the type II collagen scaffolds carrying stem cells have also been exploited for cartilage defects [133]. Consequently, we assume that the MGE based on ManNProp is also potential in cartilage repair.

## 6. Outlook and Conclusion

Metabolic glycoengineering (MGE), a technique that prospered for three decades, is now shedding new light on extensive fields. In this review, we highlighted the determinable role of glycan in regulating cell microenvironment and analyzed how MGE modifies these glycans to regulate cell fate.

Beyond those biological activities discussed in this manuscript, the MGE strategy has also been applied in a variety of biomedical fields, such as visualizing glycoconjugates for *in vivo* tracking [134], targeting agents to diagnose or kill cancer cells [135], homing of therapeutic cells [136, 137], drug delivery to promote disease recovering [138], and cell vaccine-based immunotherapies [139]. Notably, to realize the full potential of MGE, it will be necessary to explore its unveiled opportunities in regenerative medicine and bridge the gap in the current research.

In the future, we can assume the direction of MGE as (1) extend MGE application to other glycosylation pathways beyond sialic acid and discover novel metabolic precursors; (2) determine the effect of MGE in more disease models and cell types that require better regenerative distribute, such as myocardial infarction (cardiomyocytes), diabetes (pancreatic beta cells), leukemia (hematopoietic stem cells), or any other disease suitable for stem cell transplantation; (3) bioorthogonal modification of stem cells holds great prospect since the click chemistry allows more complex combination, which may lead to broader methods in altering the stem cell niche; (4) the sustainability of modified groups due to natural catabolism of glycans ought to be ameliorated; and (5) translating the current development of MGE into clinical practice has to be on its way.

In conclusion, this review summarized the MGE's application in tissue engineering and regenerative medicine, and the booming diversity of MGE ensures a broad prospect for this technique in the future.

## Figures and Tables

**Figure 1:** Interactions in the microenvironment. Cells reside in a dynamic environment consisting of ECM components, adjacent cells, mechanical forces, and various biological cues. The cell membranes offer platforms for cellular activities within their microenvironment, including molecule recognition, cell-cell interaction, and cell-matrix combination, which will, respectively, lead to different cell fates. Cell-surface glycans wrapped the membranes of cells and mediated those interactions in the microenvironment.

**Figure 2:** Overview of metabolic glycoengineering. (a) Illustration of MGE. Natural sugars are absorbed into cells and then metabolically assembled onto the cell surface as glycoconjugates (e.g., ManNAc into Neu5Ac). The analogs of metabolic precursors (ManNAc) can intercept the glycosylation pathways in cells, resulting in the submission of R-group-modified glycans and the modification of membranes. (b) Examples of MGE analogs. The analogs of MGE can be mainly classified into four catalogs: modification with aliphatic group, bioorthogonal group, thiol group, and short-chain fatty acid. The red marked text represents the R-group of different MGE analogs while the “high flux” indicates peracylated analogs with higher efficiency of modification.

## Data Availability

Data sharing is not applicable to this article as no new data was created or analyzed in this study.

## References

[1] Bacakova L., Zarubova J., Travnickova M. (2018). Stem cells: their source, potency and use in regenerative therapies with focus on adipose-derived stem cells - a review. *Biotechnology Advances*.

[2] Watt F. M., Driskell R. R. (2010). The therapeutic potential of stem cells. *Philosophical Transactions of the Royal Society B: Biological Sciences*.

[3] Discher D. E., Mooney D. J., Zandstra P. W. (2009). Growth factors, matrices, and forces combine and control stem cells. *Science*.

[4] Cuahtecontzi Delint R., Day G. J., Macalester W. J. P., Kafienah W., Xiao W., Perriman A. W. (2021). An artificial membrane binding protein-polymer surfactant nanocomplex facilitates stem cell adhesion to the cartilage extracellular matrix. *Biomaterials*.

[5] Aragona M., Dekoninck S., Rulands S. (2017). Defining stem cell dynamics and migration during wound healing in mouse skin epidermis. *Nature Communications*.

[6] Evens L., Beliën H., Deluyker D. (2020). The impact of advanced glycation end-products (AGEs) on proliferation and apoptosis of primary stem cells: a systematic review. *Stem Cells International*.

[7] Vining K. H., Mooney D. J. (2017). Mechanical forces direct stem cell behaviour in development and regeneration. *Nature Reviews. Molecular Cell Biology*.

[8] Muncie J. M., Weaver V. M. (2018). The physical and biochemical properties of the extracellular matrix regulate cell fate. *Current Topics in Developmental Biology*.

[9] Kirouac D. C., Madlambayan G. J., Yu M., Sykes E. A., Ito C., Zandstra P. W. (2009). Cell-cell interaction networks regulate blood stem and progenitor cell fate. *Molecular Systems Biology*.

[10] Zhang S. Y., Zhou Z. R., Qian R. C. (2021). Recent progress and perspectives on cell surface modification. *Chemistry, an Asian Journal*.

[11] Jing B., Gai Y., Qian R. (2021). Hydrophobic insertion-based engineering of tumor cell-derived exosomes for SPECT/NIRF imaging of colon cancer. *Journal of nanobiotechnology*.

[12] Cheng H., Byrska-Bishop M., Zhang C. T. (2012). Stem cell membrane engineering for cell rolling using peptide conjugation and tuning of cell-selectin interaction kinetics. *Biomaterials*.

[13] Sarkar D., Vemula P. K., Zhao W., Gupta A., Karnik R., Karp J. M. (2010). Engineered mesenchymal stem cells with self-assembled vesicles for systemic cell targeting. *Biomaterials*.

[14] Shi P., Ju E., Yan Z. (2016). Spatiotemporal control of cell-cell reversible interactions using molecular engineering. *Nature Communications*.

[15] Capicciotti C. J., Zong C., Sheikh M. O., Sun T., Wells L., Boons G. J. (2017). Cell-surface glyco-engineering by exogenous enzymatic transfer using a bifunctional CMP-Neu5Ac derivative. *Journal of the American Chemical Society*.

[16] Narimatsu Y., Joshi H. J., Nason R. (2019). An atlas of human glycosylation pathways enables display of the human glycome by gene engineered cells. *Molecular Cell*.

[17] Wang H., Alarcón C. N., Liu B. (2022). Genetically engineered and enucleated human mesenchymal stromal cells for the targeted delivery of therapeutics to diseased tissue. *Nature Biomedical Engineering*.

[18] Sadelain M., Rivière I., Riddell S. (2017). Therapeutic T cell engineering. *Nature*.

[19] Kuehn B. M. (2017). The promise and challenges of CAR-T gene therapy. *JAMA*.

[20] Bonifant C. L., Jackson H. J., Brentjens R. J., Curran K. J. (2016). Toxicity and management in CAR T-cell therapy. *Molecular Therapy-Oncolytics*.

[21] Csizmar C. M., Petersburg J. R., Wagner C. R. (2018). Programming cell-cell interactions through non-genetic membrane engineering. *Cell Chemical Biology*.

[22] Dennis J. W., Nabi I. R., Demetriou M. (2009). Metabolism, cell surface organization, and disease. *Cell*.

[23] Parker R. B., Kohler J. J. (2010). Regulation of intracellular signaling by extracellular glycan remodeling. *ACS Chemical Biology*.

[24] Mahal L. K., Yarema K. J., Bertozzi C. R. (1997). Engineering chemical reactivity on cell surfaces through oligosaccharide biosynthesis. *Science*.

[25] Du J., Meledeo M. A., Wang Z., Khanna H. S., Paruchuri V. D., Yarema K. J. (2009). Metabolic glycoengineering: sialic acid and beyond. *Glycobiology*.

[26] Wratil P. R., Horstkorte R., Reutter W. (2016). Metabolic glycoengineering with N-acyl side chain modified mannosamines. *Angewandte Chemie (International Ed. in English)*.

[27] Yang J. D., Nakamura I., Roberts L. R. (2011). The tumor microenvironment in hepatocellular carcinoma: current status and therapeutic targets. *Seminars in Cancer Biology*.

[28] Jones D. L., Wagers A. J. (2008). No place like home: anatomy and function of the stem cell niche. *Nature Reviews Molecular Cell Biology*.

[29] Barthes J., Özçelik H., Hindié M., Ndreu-Halili A., Hasan A., Vrana N. E. (2014). Cell microenvironment engineering and monitoring for tissue engineering and regenerative medicine: the recent advances. *BioMed Research International*.

[30] Gattazzo F., Urciuolo A., Bonaldo P. (2014). Extracellular matrix: a dynamic microenvironment for stem cell niche. *Biochimica et Biophysica Acta*.

[31] Chen C. S., Mrksich M., Huang S., Whitesides G. M., Ingber D. E. (1997). Geometric control of cell life and death. *Science*.

[32] Schlie-Wolter S., Ngezahayo A., Chichkov B. N. (2013). The selective role of ECM components on cell adhesion, morphology, proliferation and communication in vitro. *Experimental Cell Research*.

[33] Volpato F. Z., Führmann T., Migliaresi C., Hutmacher D. W., Dalton P. D. (2013). Using extracellular matrix for regenerative medicine in the spinal cord. *Biomaterials*.

[34] Gekas J., Hindié M., Faucheux N. (2004). The inhibition of cell spreading on a cellulose substrate (cuprophan) induces an apoptotic process via a mitochondria-dependent pathway. *FEBS Letters*.

[35] Frisch S., Francis H. (1994). Disruption of epithelial cell-matrix interactions induces apoptosis. *Journal of Cell Biology*.

[36] Usui A., Ko S. Y., Barengo N., Naora H. (2014). P-cadherin promotes ovarian cancer dissemination through tumor cell aggregation and tumor–peritoneum interactions. *Molecular Cancer Research*.

[37] Lairson L. L., Lyssiotis C. A., Zhu S., Schultz P. G. (2013). Small molecule–based approaches to adult stem cell therapies. *Annual Review of Pharmacology and Toxicology*.

[38] Lowe J. B. (2002). Glycosylation in the control of selectin counter-receptor structure and function. *Immunological Reviews*.

[39] Kulkarni R., Kale V. (2020). Physiological cues involved in the regulation of adhesion mechanisms in hematopoietic stem cell fate decision. *Frontiers in Cell and Development Biology*.

[40] Griffin M. E., Hsieh-Wilson L. C. (2016). Glycan engineering for cell and developmental biology. *Cell Chemical Biology*.

[41] Tian E., Ten Hagen K. G. (2009). Recent insights into the biological roles of mucin-type O-glycosylation. *Glycoconjugate Journal*.

[42] Eichler J. (2019). Protein glycosylation. *Current Biology*.

[43] Hasehira K., Hirabayashi J., Tateno H. (2017). Structural and quantitative evidence of *α*2-6-sialylated N-glycans as markers of the differentiation potential of human mesenchymal stem cells. *Glycoconjugate Journal*.

[44] Yale A. R., Nourse J. L., Lee K. R. (2018). Cell surface N-glycans influence electrophysiological properties and fate potential of neural stem cells. *Stem Cell Reports*.

[45] Zhang L., Ten Hagen K. G. (2011). The cellular microenvironment and cell adhesion: a role for O-glycosylation. *Biochemical Society Transactions*.

[46] Wilson K. M., Jagger A. M., Walker M. (2018). Glycans modify mesenchymal stem cell differentiation to impact the function of resulting osteoblasts. *Journal of Cell Science*.

[47] Ragni E., Lommel M., Moro M. (2016). Protein O-mannosylation is crucial for human mesencyhmal stem cells fate. *Cellular and Molecular Life Sciences*.

[48] Li F., Ding J. (2019). Sialylation is involved in cell fate decision during development, reprogramming and cancer progression. *Protein & Cell*.

[49] Kim S. H., Turnbull J., Guimond S. (2011). Extracellular matrix and cell signalling: the dynamic cooperation of integrin, proteoglycan and growth factor receptor. *The Journal of Endocrinology*.

[50] Almaraz R. T., Tian Y., Bhattarcharya R. (2012). Metabolic Flux Increases Glycoprotein Sialylation: Implications for Cell Adhesion and Cancer Metastasis. *Molecular & Cellular Proteomics*.

[51] Brizzi M. F., Tarone G., Defilippi P. (2012). Extracellular matrix, integrins, and growth factors as tailors of the stem cell niche. *Current Opinion in Cell Biology*.

[52] Horstkorte R., Rau K., Reutter W., Nöhring S., Lucka L. (2004). Increased expression of the selectin ligand sialyl- Lewis^x^ by biochemical engineering of sialic acids. *Experimental Cell Research*.

[53] Läubli H., Borsig L. (2010). Selectins promote tumor metastasis. *Seminars in Cancer Biology*.

[54] Bieberich E., MacKinnon S., Silva J., Yu R. K. (2001). Regulation of apoptosis during neuronal differentiation by ceramide and b-series complex gangliosides. *The Journal of Biological Chemistry*.

[55] Kontou M., Weidemann W., Bork K., Horstkorte R. (2009). Beyond glycosylation: sialic acid precursors act as signaling molecules and are involved in cellular control of differentiation of PC12 cells. *Biological Chemistry*.

[56] Kayser H., Zeitler R., Kannicht C., Grunow D., Nuck R., Reutter W. (1992). Biosynthesis of a nonphysiological sialic acid in different rat organs, using N-propanoyl-D-hexosamines as precursors. *The Journal of Biological Chemistry*.

[57] Kayser H., Ats C., Lehmann J., Reutter W. (1993). New amino sugar analogues are incorporated at different rates into glycoproteins of mouse organs. *Experientia*.

[58] Gross H. J., Brossmer R. (1988). Enzymatic introduction of a fluorescent sialic acid into oligosaccharide chains of glycoproteins. *European Journal of Biochemistry*.

[59] Gross H. J., Rose U., Krause J. M. (1989). Transfer of synthetic sialic acid analogues to N- and O-linked glycoprotein glycans using four different mammalian sialyltransferases. *Biochemistry*.

[60] Brossmer R., Gross H. J. (1994). [12] Fluorescent and photoactivatable sialic acids. *Methods in Enzymology*.

[61] Wratil P. R., Horstkorte R. (2017). Metabolic glycoengineering of sialic acid using N-acyl-modified mannosamines. *Journal of Visualized Experiments*.

[62] Keppler O. T., Herrmann M., von der Lieth C. W., Stehling P., Reutter W., Pawlita M. (1998). Elongation of the *N* -Acyl Side Chain of Sialic Acids in MDCK II Cells Inhibits Influenza A Virus Infection. *Biochemical and Biophysical Research Communications*.

[63] Templeton K., Ramos M., Rose J. (2021). Mesenchymal stromal cells regulate sialylations of N-glycans, affecting cell migration and survival. *International Journal of Molecular Sciences*.

[64] Roehlecke C., Horstkorte R., Reutter W. (2013). Stimulation of human peripheral blood mononuclear cells by the sialic acid precursor N-propanoylmannosamine. *Glycoconjugate Journal*.

[65] Hapuarachchige S., Zhu W., Kato Y., Artemov D. (2014). Bioorthogonal, two-component delivery systems based on antibody and drug-loaded nanocarriers for enhanced internalization of nanotherapeutics. *Biomaterials*.

[66] Tu Y., Dong Y., Wang K., Shen S., Yuan Y., Wang J. (2020). Intercellular delivery of bioorthogonal chemical receptors for enhanced tumor targeting and penetration. *Biomaterials*.

[67] Zhao Z., Zhang Z., Duan S. (2021). Cytosolic protein delivery via metabolic glycoengineering and bioorthogonal click reactions. *Biomaterials Science*.

[68] Fernández-Suárez M., Baruah H., Martínez-Hernández L. (2007). Redirecting lipoic acid ligase for cell surface protein labeling with small-molecule probes. *Nature Biotechnology*.

[69] Sawa M., Hsu T. L., Itoh T. (2006). Glycoproteomic probes for fluorescent imaging of fucosylated glycans in vivo. *Proceedings of the National Academy of Sciences of the United States of America*.

[70] Vocadlo D. J., Hang H. C., Kim E. J., Hanover J. A., Bertozzi C. R. (2003). A chemical approach for identifying O-GlcNAc-modified proteins in cells. *Proceedings of the National Academy of Sciences of the United States of America*.

[71] Dube D. H., Prescher J. A., Quang C. N., Bertozzi C. R. (2006). Probing mucin-type O-linked glycosylation in living animals. *Proceedings of the National Academy of Sciences of the United States of America*.

[72] Agatemor C., Buettner M. J., Ariss R., Muthiah K., Saeui C. T., Yarema K. J. (2019). Exploiting metabolic glycoengineering to advance healthcare. *Nature Reviews Chemistry*.

[73] Cheng B., Xie R., Dong L., Chen X. (2016). Metabolic remodeling of cell-surface sialic acids: principles, applications, and recent advances. *Chembiochem*.

[74] Mahal L. K., Charter N. W., Angata K., Fukuda M., Koshland D. E., Bertozzi C. R. (2001). A small-molecule modulator of poly-*α*2,8-sialic acid expression on cultured neurons and tumor cells. *Science*.

[75] Shen Y., Gao M., Ma Y. (2015). Effect of surface chemistry on the integrin induced pathway in regulating vascular endothelial cells migration. *Colloids and Surfaces. B, Biointerfaces*.

[76] Villavicencio-Lorini P., Laabs S., Danker K., Reutter W., Horstkorte R. (2002). Biochemical engineering of the acyl side chain of sialic acids stimulates integrin-dependent adhesion of HL60 cells to fibronectin. *Journal of Molecular Medicine (Berlin, Germany)*.

[77] Natunen S., Lampinen M., Suila H. (2013). Metabolic glycoengineering of mesenchymal stromal cells with N-propanoylmannosamine. *Glycobiology*.

[78] Dykstra B., Lee J., Mortensen L. J. (2016). Glycoengineering of E-selectin ligands by intracellular versus extracellular fucosylation differentially affects osteotropism of human mesenchymal stem cells. *Stem Cells*.

[79] Horstkorte R., Lee H. Y., Lucka L., Danker K., Mantey L., Reutter W. (2001). Biochemical engineering of the side chain of sialic acids increases the biological stability of the highly sialylated cell adhesion molecule CEACAM1. *Biochemical and Biophysical Research Communications*.

[80] Sampathkumar S. G., Jones M. B., Yarema K. J. (2006). Metabolic expression of thiol-derivatized sialic acids on the cell surface and their quantitative estimation by flow cytometry. *Nature Protocols*.

[81] Sampathkumar S. G., Li A. V., Jones M. B., Sun Z., Yarema K. J. (2006). Metabolic installation of thiols into sialic acid modulates adhesion and stem cell biology. *Nature Chemical Biology*.

[82] Du J., Che P. L., Wang Z. Y., Aich U., Yarema K. J. (2011). Designing a binding interface for control of cancer cell adhesion via 3D topography and metabolic oligosaccharide engineering. *Biomaterials*.

[83] Koo H., Choi M., Kim E., Hahn S. K., Weissleder R., Yun S. H. (2015). Bioorthogonal click chemistry-based synthetic cell glue. *Small*.

[84] Koo H., Hahn S. K., Yun S. H. (2016). Controlled detachment of chemically glued cells. *Bioconjugate Chemistry*.

[85] Plumet C., Mohamed A. S., Vendeuvre T., Renoux B., Clarhaut J., Papot S. (2021). Cell-cell interactions via non-covalent click chemistry. *Chemical Science*.

[86] Schmidt C., Stehling P., Schnitzer J., Reutter W., Horstkorte R. (1998). Biochemical engineering of neural cell surfaces by the synthetic N-propanoyl-substituted neuraminic acid precursor. *The Journal of Biological Chemistry*.

[87] Büttner B., Kannicht C., Schmidt C. (2002). Biochemical engineering of cell surface sialic acids stimulates axonal growth. *The Journal of Neuroscience*.

[88] Schmidt C., Ohlemeyer C., Kettenmann H., Reutter W., Horstkorte R. (2000). Incorporation of N-propanoylneuraminic acid leads to calcium oscillations in oligodendrocytes upon the application of GABA. *FEBS Letters*.

[89] Horstkorte R., Rau K., Laabs S., Danker K., Reutter W. (2004). Biochemical engineering of the N-acyl side chain of sialic acid leads to increased calcium influx from intracellular compartments and promotes differentiation of HL60 cells. *FEBS Letters*.

[90] Witzel C., Reutter W., Stark G. B., Koulaxouzidis G. (2015). N-Propionylmannosamine stimulates axonal elongation in a murine model of sciatic nerve injury. *Neural Regeneration Research*.

[91] Koulaxouzidis G., Reutter W., Hildebrandt H., Stark G. B., Witzel C. (2015). In vivo stimulation of early peripheral axon regeneration by N-propionylmannosamine in the presence of polysialyltransferase ST8SIA2. *Journal of Neural Transmission (Vienna)*.

[92] Nusse R., Clevers H. (2017). Wnt/*β*-catenin signaling, disease, and emerging therapeutic modalities. *Cell*.

[93] Du J., Agatemor C., Saeui C. T., Bhattacharya R., Jia X., Yarema K. J. (2021). Glycoengineering human neural and adipose stem cells with novel thiol-modified N-acetylmannosamine (ManNAc) analogs. *Cell*.

[94] Bagchi D. P., Nishii A., Li Z. (2020). Wnt/*β*-catenin signaling regulates adipose tissue lipogenesis and adipocyte-specific loss is rigorously defended by neighboring stromal-vascular cells. *Molecular Metabolism*.

[95] Okeley N. M., Toki B. E., Zhang X. (2013). Metabolic engineering of monoclonal antibody carbohydrates for antibody-drug conjugation. *Bioconjugate Chemistry*.

[96] Bassagañas S., Pérez-Garay M., Peracaula R. (2014). Cell surface sialic acid modulates extracellular matrix adhesion and migration in pancreatic adenocarcinoma cells. *Pancreas*.

[97] Nagasundaram M., Horstkorte R., Gnanapragassam V. S. (2020). Sialic acid metabolic engineering of breast cancer cells interferes with adhesion and migration. *Molecules*.

[98] Lo C. Y., Weil B. R., Palka B. A., Momeni A., Canty J. M., Neelamegham S. (2016). Cell surface glycoengineering improves selectin-mediated adhesion of mesenchymal stem cells (MSCs) and cardiosphere-derived cells (CDCs): pilot validation in porcine ischemia-reperfusion model. *Biomaterials*.

[99] Reily C., Stewart T. J., Renfrow M. B., Novak J. (2019). Glycosylation in health and disease. *Nature Reviews. Nephrology*.

[100] Kim E. J., Sampathkumar S. G., Jones M. B. (2004). Characterization of the metabolic flux and apoptotic effects of O-hydroxyl- and N-acyl-modified N-acetylmannosamine analogs in Jurkat cells. *Journal of Biological Chemistry*.

[101] Almaraz R. T., Aich U., Khanna H. S. (2012). Metabolic oligosaccharide engineering with N-acyl functionalized ManNAc analogs: cytotoxicity, metabolic flux, and glycan-display considerations. *Biotechnology and Bioengineering*.

[102] Mathew M. P., Tan E., Saeui C. T. (2015). Metabolic glycoengineering sensitizes drug-resistant pancreatic cancer cells to tyrosine kinase inhibitors erlotinib and gefitinib. *Bioorganic & Medicinal Chemistry Letters*.

[103] Mao D., Zhang C., Kenry (2020). Bio-orthogonal click reaction-enabled highly specific in situ cellularization of tissue engineering scaffolds. *Biomaterials*.

[104] Oh B., Swaminathan V., Malkovskiy A., Santhanam S., McConnell K., George P. M. (2020). Single-cell encapsulation via click-chemistry alters production of paracrine factors from neural progenitor cells. *Advanced Science*.

[105] Elmouelhi N., Aich U., Paruchuri V. D. P. (2009). Hexosamine template. A platform for modulating gene expression and for sugar-based drug discovery. *Journal of Medicinal Chemistry*.

[106] Nagaoka I., Igarashi M., Sakamoto K., Kim S.-K. (2012). Chapter 22- Biological activities of glucosamine and its related substances. *Advances in Food and Nutrition Research*.

[107] Li T., Liu B., Chen K., Lou Y., Jiang Y., Zhang D. (2020). Small molecule compounds promote the proliferation of chondrocytes and chondrogenic differentiation of stem cells in cartilage tissue engineering. *Biomedicine & Pharmacotherapy*.

[108] Derfoul A., Miyoshi A. D., Freeman D. E., Tuan R. S. (2007). Glucosamine promotes chondrogenic phenotype in both chondrocytes and mesenchymal stem cells and inhibits MMP-13 expression and matrix degradation. *Osteoarthritis and Cartilage*.

[109] Khoo M. L. M., McQuade L. R., Smith M. S. R., Lees J. G., Sidhu K. S., Tuch B. E. (2005). Growth and differentiation of embryoid bodies derived from human embryonic stem cells: effect of glucose and basic fibroblast growth factor1. *Biology of Reproduction*.

[110] Hwang N. S., Varghese S., Theprungsirikul P., Canver A., Elisseeff J. (2006). Enhanced chondrogenic differentiation of murine embryonic stem cells in hydrogels with glucosamine. *Biomaterials*.

[111] Ma Y., Zheng W., Chen H. (2018). Glucosamine promotes chondrocyte proliferation via the Wnt/*β*-catenin signaling pathway. *International Journal of Molecular Medicine*.

[112] Poustie M. W., Carran J., McEleney K., Dixon S. J., Anastassiades T. P., Bernier S. M. (2004). N-butyryl glucosamine increases matrix gene expression by chondrocytes. *The Journal of Pharmacology and Experimental Therapeutics*.

[113] Silbert J. E. (2009). Dietary glucosamine under question. *Glycobiology*.

[114] Henrotin Y., Mobasheri A., Marty M. (2012). Is there any scientific evidence for the use of glucosamine in the management of human osteoarthritis?. *Arthritis Research & Therapy*.

[115] Marcu B. K., Otero M., Olivotto E., Maria Borzi R., Goldring B. M. (2010). NF-kappaB signaling: multiple angles to target OA. *Current Drug Targets*.

[116] Campbell C. T., Aich U., Weier C. A. (2008). Targeting pro-invasive oncogenes with short chain fatty acid-hexosamine analogues inhibits the mobility of metastatic MDA-MB-231 breast cancer cells. *Journal of Medicinal Chemistry*.

[117] Coburn J. M., Wo L., Bernstein N. (2013). Short-chain fatty acid-modified hexosamine for tissue-engineering osteoarthritic cartilage. *Tissue Engineering. Part A*.

[118] Coburn J. M., Bernstein N., Bhattacharya R., Aich U., Yarema K. J., Elisseeff J. H. (2013). Differential response of chondrocytes and chondrogenic-induced mesenchymal stem cells to C1-OH tributanoylated N-acetylhexosamines. *PLoS One*.

[119] Kim C., Jeon O. H., Kim D. H. (2016). Local delivery of a carbohydrate analog for reducing arthritic inflammation and rebuilding cartilage. *Biomaterials*.

[120] Henry N., Clouet J., le Bideau J., le Visage C., Guicheux J. (2018). Innovative strategies for intervertebral disc regenerative medicine: from cell therapies to multiscale delivery systems. *Biotechnology Advances*.

[121] Binch A. L. A., Fitzgerald J. C., Growney E. A., Barry F. (2021). Cell-based strategies for IVD repair: clinical progress and translational obstacles. *Nature Reviews Rheumatology*.

[122] Clarke L. E., McConnell J. C., Sherratt M. J., Derby B., Richardson S. M., Hoyland J. A. (2014). Growth differentiation factor 6 and transforming growth factor-beta differentially mediate mesenchymal stem cell differentiation, composition, and micromechanical properties of nucleus pulposus constructs. *Arthritis Research & Therapy*.

[123] Zhou X., Wang J., Huang X. (2018). Injectable decellularized nucleus pulposus-based cell delivery system for differentiation of adipose-derived stem cells and nucleus pulposus regeneration. *Acta Biomaterialia*.

[124] Du Y., Wang Z., Wu Y., Liu C., Zhang L. (2021). Intervertebral Disc Stem/Progenitor Cells: A Promising “Seed” for Intervertebral Disc Regeneration. *Stem Cells International*.

[125] Wang J., Tao Y., Zhou X. (2016). The potential of chondrogenic pre-differentiation of adipose-derived mesenchymal stem cells for regeneration in harsh nucleus pulposus microenvironment. *Experimental Biology and Medicine (Maywood, N.J.)*.

[126] Kregar Velikonja N., Urban J., Fröhlich M. (2014). Cell sources for nucleus pulposus regeneration. *European Spine Journal*.

[127] Chooi W. H., Chew S. Y. (2019). Modulation of cell-cell interactions for neural tissue engineering: potential therapeutic applications of cell adhesion molecules in nerve regeneration. *Biomaterials*.

[128] Zhou X., Wang J., Fang W. (2018). Genipin cross-linked type II collagen/chondroitin sulfate composite hydrogel- like cell delivery system induces differentiation of adipose-derived stem cells and regenerates degenerated nucleus pulposus. *Acta Biomaterialia*.

[129] Zhou X., Ma C., Hu B. (2018). FoxA2 regulates the type II collagen-induced nucleus pulposus-like differentiation of adipose-derived stem cells by activation of the Shh signaling pathway. *The FASEB Journal*.

[130] Ying L., Liang C., Zhang Y. (2022). Enhancement of nucleus pulposus repair by glycoengineered adipose-derived mesenchymal cells. *Biomaterials*.

[131] Xing H., Lee H., Luo L., Kyriakides T. R. (2020). Extracellular matrix-derived biomaterials in engineering cell function. *Biotechnology Advances*.

[132] Liu W., Xu B., Xue W. (2020). A functional scaffold to promote the migration and neuronal differentiation of neural stem/progenitor cells for spinal cord injury repair. *Biomaterials*.

[133] Kilmer C. E., Battistoni C. M., Cox A., Breur G. J., Panitch A., Liu J. C. (2020). Collagen type I and II blend hydrogel with autologous mesenchymal stem cells as a scaffold for articular cartilage defect repair. *ACS Biomaterials Science & Engineering*.

[134] Lim S., Yoon H. Y., Jang H. J. (2019). Dual-modal imaging-guided precise tracking of bioorthogonally labeled mesenchymal stem cells in mouse brain stroke. *ACS Nano*.

[135] Wang X., Lang S., Tian Y. (2020). Glycoengineering of natural killer cells with CD22 ligands for enhanced anticancer immunotherapy. *ACS Central Science*.

[136] Donnelly C., Dykstra B., Mondal N. (2018). Optimizing human Treg immunotherapy by Treg subset selection and E-selectin ligand expression. *Scientific Reports*.

[137] Robinson S. N., Simmons P. J., Thomas M. W. (2012). Ex vivo fucosylation improves human cord blood engraftment in NOD-SCID IL-2R*γ*^null^ mice. *Experimental Hematology*.

[138] Malicdan M. C., Noguchi S., Tokutomi T. (2012). Peracetylated *N* -Acetylmannosamine, a Synthetic Sugar Molecule, Efficiently Rescues Muscle Phenotype and Biochemical Defects in Mouse Model of Sialic Acid-deficient Myopathy. *The Journal of Biological Chemistry*.

[139] Au K. M., Medik Y., Ke Q., Tisch R., Wang A. Z. (2021). Immune checkpoint-bioengineered beta cell vaccine reverses early-onset type 1 diabetes. *Advanced Materials*.

